# Bayesian Shared Frailty Models for Time to First Birth of Married Women in Ethiopia: Using EDHS 2016

**DOI:** 10.1155/2022/5760662

**Published:** 2022-08-04

**Authors:** Kenaw Derebe Fentaw, Setegn Muche Fenta, Hailegebrael Birhan Biresaw, Setegn Bayabil Agegn, Mitiku Wale Muluneh

**Affiliations:** Department of Statistics, Debre Tabor University, Debre Tabor, Ethiopia

## Abstract

**Introduction:**

The primary effect of the fertility process is the birth of the first child. The ages at which women establish marital union and give their first birth depend on and result in varying demographic features. This research demonstrates how to examine the effect of numerous factors on married women's delay to first birth in Ethiopia using Bayesian parametric models with gamma shared frailty distribution.

**Methods:**

This study analyzed data from the 2016 EDHS on factors related to the time of married women to first birth. A sample of 8810 married women from all parts of Ethiopia participated in the study. The Akaike information criterion (AIC) and Bayesian information criterion (BIC) were used to compare several parametric models with gamma shared frailty distributions to find the best model (BIC). Finally, when the prior data was taken into account, the chosen model was proven to be accurate (Bayesian approach).

**Results:**

The median survival time for the first birth after marriage is 24 years (95% CI; 23.4, 25.3). The result shows that the place of residence, the access to media, the level of education of the mother, the education level of the husband, the use of the head of the contraceptives, and the sex of the household are statistically associated with the time to first birth of married women. The Weibull-gamma shared frailty model under the Bayesian approach was found to be the best model that fit the time to first birth data in this study. The result also showed that there is heterogeneity between regions of married women.

**Conclusion:**

To slow the increase in the Ethiopian population, families must be taught how to use contraception, and rural populations must be educated on the necessity of increasing the length of the first birth gap rather than encouraging early marriage. In general, attempts to reduce fertility by raising the age of the first marriage must consider the social and cultural settings in which marriage takes place. On the other hand, the campaign against early marriage should focus on the sociocultural, physiological, and psychological effects, as well as the reduction of reproduction.

## 1. Background

The primary effect of the fertility process is the birth of the first child [1]. The ages at which women establish marital union and give their first birth depend on and result in varying demographic characteristics [2]. Every year, between the ages of 15 and 19, approximately 16 million young girls give birth. Young mothers are responsible for roughly one in every ten childbirths worldwide, with developing countries accounting for 95% of this [3]. Adolescent fertility, especially among the youngest age groups, poses serious health hazards to both the mother and the child [4–6]. The health and social causes of early-age pregnancy and childbearing are well documented, and they become major issues for the well-being of a mother and her child [7]. In the poorest parts of the world, 20% of females give birth before 18 years old, and in Kenya, this number jumps to more than a third (35%) [8]. Furthermore, women less than 15 years are five times higher chance to die, and those between the ages of 15 and 19 are twice as likely to die during pregnancy or childbirth as those between the ages of 20 and 24 [8, 9]. While sub-Saharan African countries dropped their teenage birth rate from 140 to 101 births per 1000 women aged 15–19 years over the Millennium Development Goals era (1990–2015), other regions such as South Asia, North Africa, and the Middle East saw far greater reductions [10]. In 2013, Nigeria's median age at the first birth was 20 years [11]. More than a third (34%) of Ethiopian women aged 20 to 49 years give birth before the age of 18 years and 54% at the age of 20 [12]. The high frequency of poor mother-and-child health in third-world countries can be attributed to several variables. Deep-seated sociocultural and spiritual practices, illiteracy, and low income are all part of this [11, 13, 14]. Socioeconomic characteristics were consistently identified as a predictor of age at the first birth. Many studies have shown that women with no or low levels of education had a higher chance of having their first child at a younger age than women with higher levels of education [15–17]. A study carried out in Nigeria on Bayesian semiparametric multilevel survival modelling of age at the first birth showed that variation in age at the first birth in Nigeria is determined more by individual households than by community and that substantial geographical variations exist in timing of the first birth [18]. Even though the age at which a child is born has a significant impact on maternal and infant survival, both individual and cumulative levels of fertility, and comprehensive consequences for women's roles and social changes in general, there are few studies on this topic in Ethiopia on adolescent pregnancy [19] and age at first birth after marriage [20]. However, those studies did not consider unobserved heterogeneity (shared frailty). If the data come from different groups or the nature of the data has repeated measures, heterogeneity between individuals should be taken into account [21]. Numerous issues could arise if heterogeneity is ignored, including an overestimation of the relative hazard rate, inaccurate estimates of the regression coefficients, and a tendency for the regression parameter estimate to approach zero [21]. Frailty provides a more precise estimate of the parameters compared to standard AFT models [22].

In addition, Bayesian approaches have recently been employed as the best method over classical approaches in numerous research investigations, particularly in the field of medicine. One of the problems is that traditional methods rely on asymptotic considerations that are usually only true for large datasets [23]. In the Bayesian approach, no assumption is made as to the shape of the percentile distribution; rather, the data themselves specify the distribution and the Bayesian approach has the possibility of improving the precision of the results by introducing external information in terms of the a priori distribution [23]. Understanding the time and factors that influence the first birth in the country would aid in the development of effective measures to improve mother and child health. Thus, taking into account the aforementioned limitations, this study is meant to estimate the time to first birth and find predictors among all married women in Ethiopia using a Bayesian approach while accounting for random impact (shared frailty) between regions of Ethiopia.

## 2. Methods

### 2.1. Study Area

This research was conducted in Ethiopia, which is Africa's second most populated country, after Nigeria, and is located in the Horn of Africa. Ethiopia has nine regional states (Tigray, Afar, Amhara, Oromiya, Somali, Benishangul-Gumuz, Southern Nations Nationalities and People (SNNP), Gambela, and Harari), as well as two city governments (Addis Ababa and Dire Dawa) [24].

### 2.2. Study Design

Enumeration areas (EAs) were the sampling units for the first stage of the 2016 EDHS sample, which was chosen using a stratified two-stage cluster design. During the 2007 census, each kebele (ward) was partitioned into census enumeration areas (EAs) to make the census easier to administer. There were 645 EAs in the sample, with 187 in urban regions and 437 in rural areas. The second stage of the sampling involved households. The interviews were open to all women aged 15 to 49 years. Individual interviews were done with 16,583 eligible women from the interviewed households; complete interviews were conducted with 15,683 [25]. In the current study, 8810 married women from nine regions and two city administrations were included (Figure 1).

### 2.3. Study Population

The current study used married women data from the Ethiopian Demographic and Health Surveys (EDHS) conducted in 2016.

### 2.4. Variables Included in the Study

#### 2.4.1. Dependent Variable

The response variable is the time to first birth of married women in Ethiopia. It is measured as the length of time from birth to the age at the first birth, which is measured in years.

#### 2.4.2. Explanatory Variables

The expected explanatory variables included socioeconomic, demographic, health, and environmental factors (Table 1).

### 2.5. Statistical Analysis

After obtaining the consent letter for use of the measured DHS, the dataset was acquired through the website https://dhsprogram.com. A data extraction technique was used to extract variables from the EDHS 2016 dataset for children and individual women. The study population was characterized using descriptive measures like graphs and frequency tables after editing and coding. The Kaplan-Meier (K-M) and the log-rank test were calculated to show the time of the first birth and to compare the survival time between covariates, respectively. We first analyzed our data using Cox proportional hazard [26], accelerated failure time [26], and parametric shared frailty models. Then, using AIC and BIC, the best model was selected. Finally, the Bayesian parametric gamma shared frailty model was fitted, and the best model was selected using DIC criteria. Data were entered and cleaned using SPSS-22 and analyzed using WinBugs1.4.

### 2.6. Survival Analysis

Survival analysis is a set of statistical processes for data analysis for which the outcome variable of interest is the time until an event occurs. By the time, this means year, month, week, or days from the beginning of follow-up of an individual until an event occurs. By event, it means death, disease incidence, relapse from remission, recovery (e.g., return to work), or any designated experience of interest that may happen to an individual. Despite these, survival models have a long history in the biostatistical and medical literature [27].

### 2.7. The Cox Proportional Hazard Model

The Cox proportional hazards regression model is a model that assumes that the log of hazard rate is additively related to a function of covariates or the hazard rate is related multiplicatively to a function of covariates [26]. This model presents an equation for the hazard at time *t* for an individual with a particular collection of explanatory factors indicated by *X*, and it is usually expressed as

(1) $$\begin{array}{c} h\left(t,X,\beta \right)=h_{0}\left(t\right)\exp\left(X\beta \right), \end{array}$$

where *h*_0_(*t*) is the baseline hazard function at time *t*, *X* is the vector of values of the explanatory variables, and *β* = (*β*_1_, *β*_2_, ⋯, *β*_*k*_) is the vector of unknown regression parameters that are assumed to be the same for all individuals in the study, which measures the influence of the covariate on the survival experience.

### 2.8. Parametric Survival Model

If our survival time follows a specified probability distribution, we apply parametric survival models, and the parameters of that distribution depend on covariates. Among the popular parametric survival models, some of them are exponential, Gompertz, Weibull, log-normal, and log-logistic.

### 2.9. Exponential Distribution

The simplest model for the hazard function is to assume that it is constant over time. The hazard of death at any time after the time origin of the study is then the same irrespective of the time elapsed. This famous property of the exponential distribution is known as “loss of memory” which requires that the age of the person does not affect future survival. Let *t* be the survival time that follows exponential distribution with parameter *λ*. Then, the pdf of *t* is

(2) $$\begin{array}{c} f\left(x\right)=\lambda e^{-\lambda t},\;t>,\lambda >0, \end{array}$$

and *h*(*t*) = *λ*.

### 2.10. Gompertz Distribution

The Gompertz model has found application in demography and the biological sciences. The probability density function of the Gompertz distribution is given by

(3) $$\begin{array}{c} f\left(t\right)=\lambda e^{\theta t}\exp\left[\frac{\lambda }{\theta }\left(1-e^{\theta t}\right)\right],\;t>0,\lambda >0, \end{array}$$

*h*(*t*) = *λe*^*θt*^ and exp[(*λ*/*θ*)(1 − *e*^*θt*^)].

### 2.11. Weibull Distribution

Weibull distributions are parameterized as both proportional hazard (pH) and accelerated failure time (AFT) models. The Weibull distribution is suitable for modeling data with monotone hazard rates that increase or decrease exponentially over time. For Weibull regression, *λ* is the scale parameter and *γ* is a shape parameter, and its probability distribution function is given by

(4) $$\begin{array}{c} f\left(\text{t}\right)=\lambda \gamma {\text{t}}^{\gamma -1}e^{-\lambda t\gamma },\;\lambda ,\gamma >0, \end{array}$$

*S*(t) = *e*^−*λtγ*^ and *h*(t) = *λγt*^*γ*−1^.

### 2.12. The Log-Logistic Distribution

One limitation of the Weibull hazard is that it is a monotonic function of time. However, situations can arise in which the hazard function changes direction. In this situation, log-logistic is a preferable model.

(5) $$\begin{array}{c} f\left(\text{t}\right)=\frac{e^{\theta }{kt}^{k-1}}{{\left(1+e^{\theta }t^{k}\right)}^{2}}, \end{array}$$

*h*(t) = *e*^*θ*^*kt*^*k*−1^/(1 + *e*^*θ*^*t*^*k*^)^2^ for 0 ≤ *t* < ∞, *k* > 0 and *S*(*t*) = 1/(1 + *e*^*θ*^*t*^*k*^).

Note that the hazard function decreases monotonically if *K* ≤ 1, but if *K* > 1, the hazard has a single mode.

### 2.13. The Log-Normal Distribution

The log-normal distribution is also defined for random variables that take positive values and so may be used as a model for survival data. A random variable *T* is said to have a log-normal distribution with parameters *μ* and *δ*log*T*, and it has a normal distribution with *μ* and variance *σ*. The probability density function of *T* is given by

(6) $$\begin{array}{c} f\left(\text{t}\right)=\frac{1}{\delta \sqrt{2\pi }}t^{-1}\exp\left(\frac{{\left(-\log t‐\mu \right)}^{2}}{2\delta^{2}}\right),\;0\leq t<\infty ,\delta >0. \end{array}$$

The survivor function of the log-normal distribution is *S*(*t*) = 1 − *Φ*((log*t*‐*μ*)/*δ*) where *Φ*(.) is the standard normal distribution function given by *Φ*(*z*) = (1)(2*π*)^1/2^∫_−∞_^*z*^exp(−*u*^2^/2)*du* and *h*(*t*) = *f*(*t*)/*S*(*t*).

### 2.14. Parametric Shared Frailty Model

The multivariate or shared frailty model is a conditional independence model in which frailty is common to all subjects in a cluster. In this study, the clusters are regions. The concept of frailty provides a suitable way to introduce random effects into the model to account for association and unobserved heterogeneity. In its simplest form, frailty is an unobserved random factor that modifies multiplicatively the hazard function of an individual or cluster of individuals. [28] introduced the term frailty, and [29] promoted the model by its application to the multivariate situation on the incidence of chronic diseases in families. There are different frailty distributions such as gamma [22], inverse Gaussian [30], log-normal [31], and positive stable [32]. However, the gamma distribution is the most common and widely used in the literature for determining the frailty effect, which acts multiplicatively on the baseline hazard [30, 33].

Let us have *k* observations and *i* subgroups (regions). Each region consists of *n*_*i*_ observations and ∑_*i*=1_^*r*^*ni* = *n*, where *n* is the total sample size. The hazard rate for the *k*^th^ individual in the *i*^th^ region is given by

(7) $$\begin{array}{c} h_{ik}\left(t\right)=h_{0}\left(t\right)\exp\left(X_{ik}^{\prime }\beta +Zi\right),\;i=1,2,\cdots r,k=1,2,\cdots n_{i}. \end{array}$$

Here, frailty *Z* is a random variable varying over the population decrease (*Z* < 1) or increases (*Z* > 1) the individual risk. The most important point here is that the frailty is unobservable. The respective survival function *S*, describing the fraction of surviving individuals in the study population, is given by *S*(*t*, *X*, *Z*) = exp(−*Z*∫_0_^*t*^*ho*(*u*)*du*exp(*Xβ*)). The cumulative hazard function is given by *H*(t) = ∫_0_^*t*^*h*_0_(*u*)*du*.

The main assumption of a shared frailty model is that all individuals in region *i* share the same value of frailty *Z*_*i*_ (*i* = 1, 2, 3, ⋯, *m*), and this is why the model is called the shared frailty model. In our study, the women assumed to share some common frailty in the region. The shared frailty (random) effect *Z*_*i*_ follows a gamma distribution with mean one and variance *θ*, as defined in the density function in equation (6).

(8) $$\begin{array}{c} f_{z}\left(Z\right)=\frac{z^{\left(1-\theta \right)/\theta }\exp\left(-\text{z}/\theta \right)}{\theta^{1/\theta }\Gamma \left(1/\theta \right)},\;\theta >0, \end{array}$$

where *θ* > 0 indicates the presence of heterogeneity. Therefore, the high values of *θ* reflect a greater degree of heterogeneity among regions of pregnant women and a stronger association within regions.

The associations within group members (regions) are measured by Kendall's, and gamma frailty distribution is given by

(9) $$\begin{array}{c} \Gamma =\frac{\theta }{\theta +2}\in \left(0,1\right). \end{array}$$

### 2.15. Bayesian Parametric Gamma Shared Frailty Models

In the Bayesian approach, the critical issue is identifying the prior distribution for each parameter in the model to get a best-fit posterior distribution. The prior distribution is a probability distribution that represents the prior information associated with the parameter of interest. In this study, we used noninformative priors for all parameters of interest.

Let *δ*_*ij*_ denote the censoring indicator variable, taking value 1 if the *j*^th^ subject (*j* = 1, 2, ⋯, *m*_*i*_) of the *i*^th^ cluster (*i* = 1, 2, ⋯, *n*) fails and 0 otherwise; *T* = (*t*_11_, *t*_12,._..,*t*_*nm*_)′ and *X* = (*x*_1_, *x*_2_, ⋯, *x*_*n*_), where *x*_*i*_ is the *m* × *n* matrix of covariates. Let *D* = (*X*, *T*, *δ*_*ij*_, *Z*) denote the complete data, and let *D*_obs_ = (*X*, *T*, *δ*_*ij*_) denote the observed data. Here, we only allow for the right-censored survival data and assume that the censoring is noninformative. The complete data likelihood is given:

(10) $$\begin{array}{c} L\left(\beta ,\theta ,\frac{\wedge_{0}}{D}\right)=\overset{m}{\underset{j=1}{\prod }}\overset{n}{\underset{i=1}{\prod }}f{\left({\frac{t_{ij}}{x}}_{i},z\right)}^{\delta_{jj}}*S{\left(\frac{t_{jj}}{x_{i}},z\right)}^{1-\delta_{jj}}=\overset{m}{\underset{j=1}{\prod }}\overset{n}{\underset{i=1}{\prod }}h{\left(\frac{t_{ij}}{z_{ij}}\right)}^{\delta_{j}}*S\left(\frac{t_{jj}}{z_{ji}}\right),\text{where }h\left(\frac{t}{z},x\right)=h_{0}\left(t\right)e^{\left(\beta xi+zj\right)},S\left(\frac{t}{x_{i}},z_{i}\right)=\text{Exp}-\left(\Delta_{0}\left(t\right)e^{\left(\beta x+z\right)}\right),\Delta_{0}=\int_{0}^{t}h\left(u\right)du,\\ \text{i}.\text{e}.,L\left(\beta ,\theta ,\frac{\wedge_{0}}{D}\right)=\overset{m}{\underset{j=1}{\prod }}\overset{n}{\underset{i=1}{\prod }}{\left(h_{0}\left(t\right)\exp^{\left(\beta x+z\right)}\right)}^{\delta_{j}}*\left[\text{Exp}-\left(\Delta_{0}\left(t\right)e^{\left(\beta x+z\right)}\right)\right], \end{array}$$

where *β*, ∧_0_, and *θ* are the regression coefficient, the baseline distribution parameters, and the gamma frailty distribution parameters, respectively.

Because the observed data likelihood is simply too intricate to work with, evaluating the joint posterior distribution analytically is challenging. We employ the Gibbs sampler to obtain samples from the joint posterior distribution to avoid this problem.

(11) $$\begin{array}{c} L\left(\beta ,\wedge_{0},\frac{\theta }{D_{\text{obs}}}\right)=\overset{m}{\underset{j=1}{\prod }}\overset{n}{\underset{i=1}{\prod }}\int_{0}^{\infty }L\left(\beta ,\wedge_{0},\frac{\theta }{D}\right)f\left(z\right)dz,\;\text{where }f_{z}\left(Z\right)=\frac{z^{\left(1-\theta \right)/\theta }\exp\left(-z/\theta \right)}{\theta^{1/\theta }\Gamma \left(1/\theta \right)},\theta >0. \end{array}$$

### 2.16. Prior Distributions

In Bayesian inference, prior elicitation may be the most important factor. The prior distributions for each parameter in the model must be specified first before we can do data analysis from a Bayesian perspective. We want our data information to dominate the prior distribution by assuming suitably noninformative priors for all parameters in this model because we have little prior information for all parameters to be estimated. We used independent imprecise normal priors with a mean of 0 and a variance of 1∗10^5^ for all regression coefficients. A gamma distribution with shape parameter 1 and scale parameter 0.001 (with mean 1000 and variance 1∗10^6^) is used to supply noninformative priors to the scale and shape parameters in the model. We use the hazy proper gamma prior distribution with shape parameter 0.001 and scale parameter 0.001 for their reciprocals for the shared frailty parameter (precision parameters for the random effects).

### 2.17. Posterior Distributions

By multiplying the prior distribution across all parameters *φ*, by the entire likelihood function *L*(*ϕ*/*y*), the posterior distribution is derived. The posterior distribution of the model created informs all Bayesian inferential judgments. The inference is carried out by sampling from a posterior distribution until the posterior distribution converges. The main drawback of the Bayesian technique is that, in most circumstances, the whole form of the posterior distribution cannot be derived in a closed form, implying that the posterior density may not belong to the standard distribution. This is a difficult problem to solve. MCMC simulations will be used to solve these challenges.

We start with the joint density function of observable information *Y* and latent information *Z* to obtain the posterior densities.

(12) $$\begin{array}{c} f\left(\frac{y}{\phi }\right),\text{with }\varphi =\left(\beta ,\theta ,\wedge_{0}\right). \end{array}$$

Then, we will pretend that *φ* is a random variable with a prior distribution defined by *π*(*ϕ*). The posterior distribution, which is derived using Bayes' theorem, is then used to make inferences. The posterior distribution *ϕ* is then calculated as follows: *f*(*ϕ*/*y*) = *L*(*ϕ*/*y*)*π*(*ϕ*)/*f*(*y*) = *f*(*y*/*ϕ*)*π*(*ϕ*)/*f*(*y*), where *f*(*y*) = ∫*L*(*ϕ*/*y*)*π*(*ϕ*)*dφ* is a normalizing factor (constant). Thus, we have *f*(*φ*/*y*) ∝ *L*(*ϕ*/*y*)*π*(*ϕ*).

The joint posterior density function of a parameter at a certain failure time is derived by using this expression and assuming independence between the prior density functions of the parameters.

(13) $$\begin{array}{c} \pi \left(\phi =\theta ,\beta ,\frac{\wedge_{0}}{t}\right)\propto L\left(\phi =\frac{\left(\theta ,\beta ,\wedge_{0}\right)}{D_{\text{obs}}}\right)g_{1}\left(\theta \right)*\overset{k}{\underset{i=1}{\prod }}g_{2i}\left(\wedge_{0}\right)*\prod \pi_{i}\left(\beta_{i}\right), \end{array}$$

where *g*_*i*_(.) indicates the prior density function with known hyperparameters of the corresponding argument for baseline parameters and frailty variance. *π*_*i*_(*β*_*i*_) is the prior density function for the regression coefficients *β*_*i*_ for *i* = 1, 2, ⋯, *r*. Also, the equation gives the likelihood function:

(14) $$\begin{array}{c} L\left(\phi =\frac{\left(\theta ,\beta ,\wedge_{0}\right)}{D_{\text{obs}}}.\right. \end{array}$$

The graphical representation of multivariate distributions well known in connection with for models high dimensional contingency tables and Bayesian inference in expert system [34]. Graph theory is also useful in the study of Markov random fields, which are important in statistical mechanics and, more recently, spatial statistics and image analysis. The general layout of this research is presented in Figure 2.

### 2.18. MCMC Estimation Methods

The Bayesian approach, often known as “full probability modeling,” adds probability theory to a model formed from substantive information and can, in theory, deal with truly complex circumstances. However, it must be emphasized that the computations may be challenging, with the specific challenge being the integration required to determine the posterior distributions of the quantities of interest when nonstandard prior distributions are utilized in the model. For many years, these integration issues limited Bayesian applications to rather simple cases. However, there has been a lot of improvement recently in Bayesian computation methods, which generally take advantage of modern computing power to do simulations known as Markov Chain Monte Carlo (MCMC) approaches. Although the shape of the posterior distribution of interest has no known algebraic form, the MCMC simulation performs the integration numerically rather than analytically by sampling from the posterior distribution of interest [34]. All posterior summary statistics will be generated as a result of this procedure (approximately). The most commonly used algorithms in MCMC applications are of two types, and they are the Metropolis algorithm and the Gibbs sampler.

### 2.19. Gibbs Sampler

The Gibbs sampler is an algorithm that sequentially generates samples from a joint distribution of two or more random variables. The sampler is frequently utilized:

- The joint distribution *π*(*θ*/*x*) is not known explicitly
- The full conditional distribution of each parameter (*π*(*θ*_*i*_/*θ*_*j*_, *X*), *i* ≠ *j*) is not known

#### 2.19.1. Algorithm of the Gibbs Sampler

(1) Choose an arbitrary initial value of *θ*^(0)^ = {*θ*_1_^(0)^, *θ*_2_^(0)^, *θ*_3_^(0)^, ⋯⋯, *θ*_*k*_^(0)^}
(2) For *i* = 0, 1, 2, ⋯*N* − 1, generate each component of *θ* as follows:
  - Draw *θ*_1_^(*i* + 1)^ from *π*(*θ*_1_/*θ*_2_^*i*^, *θ*_3_^*i*^, ⋯, *θ*^*k*^_*i*_, *X*, *Y*)
  - Draw *θ*_2_^(*i* + 1)^ from *π*(*θ*_2_/*θ*_1_^(i + 1)^, *θ*_3_^*i*^, ⋯, *θ*^*k*^_*i*_, *X*, *Y*)
  - Draw *θ*_3_^(i + 1)^ from *π*(*θ*_3_/*θ*_1_^(*i* + 1)^, *θ*_2_^(*i* + 1)^, ⋯, *θ*^*k*^_*i*_, *X*, *Y*)
  - ⋯
  - Draw *θ*_*k*_^(i + 1)^ from *π*(*θ*_*k*_/*θ*_1_^(*i* + 1)^, *θ*_2_^(*i* + 1)^, ⋯, *θ*^*k*^^+1^_*i*−1_, *X*, *Y*)
(3) Repeat step 2 convergence
(4) Return *θ*^(*b* + 1)^ = {*θ*_1_^(*b* + 1)^, *θ*_2_^(*b* + 2)^, *θ*_3_^(*b* + 3)^, ⋯, *θ*_*k*_^(*b* + 1)^}

The standard deviations offer measures of precision, whereas the means of the posterior samples provide point estimates for the model parameters. Along with estimating precision, the 95 percent intervals provide an alternative indicator of the covariates' influence. The difference between the mean of the sampled values (which we use as our posterior mean estimate for each parameter) and the true posterior mean is calculated as the MC error. As a general rule, the simulation should be run until the Monte Carlo error for each parameter of interest is less than 5% of the sample standard deviation.

### 2.20. Model Selection Criterion by the Bayesian Approach

Computing posterior model probabilities is a typical method for comparing Bayesian models. We employ the Akaike information criterion (AIC), the Bayesian information criterion (BIC), the deviance information criterion (DIC), and the Bayes factor to compare the proposed models. These are the most prevalent Bayesian model evaluation techniques.

Given a class of competing models for a dataset, Akaike (1973) proposed that the model that minimizes be chosen.

(15) $$\begin{array}{c} \text{AIC}=D\left(\hat{\theta }\right)+2P, \end{array}$$

where *P* is the number of model parameters. $D\;\left(\hat{\theta }\right)$ is a deviation estimate based on the posterior mean, which is equal to $\hat{\;\theta }=E\;\left(\theta /\text{data}\right)$. The deviation is equal to $\hat{\theta }=-2\;\log\;L\left(\theta \right)$, where *L*(*θ*) is the likelihood function of the model and *θ* is a vector of unknown parameters of the model.

Schwarz proposed the Bayesian information criterion (BIC) (1978). [35, 36] have [33] shown that, even asymptotically, AIC tends to overstate the number of parameters required. According to the Schwarz criterion, the model that minimizes has the best posterior probability.

(16) $$\begin{array}{c} \text{BIC}=D\left(\hat{\theta }\right)+p\log\left(n\right). \end{array}$$

The number of observations, or sample size, is denoted by the letter *n*. [34] introduces DIC, a generalization of AIC, which is defined as $\text{DIC}=D\left(\hat{\theta }\right)+2p_{d}$, where *p* (*d*) is the difference between the posterior mean of the deviation and the deviance of the posterior mean of the parameters of interest, i.e., $PD=\bar{D}-D\left(\hat{\theta }\right)$ and $\bar{D}=E\left(\theta /\text{data}\right)$. Models with lower AIC, BIC, and DIC values are favored.

## 3. Results

### 3.1. Descriptive Statistics

The descriptive statistics of the variables in Table 2 show that a total of 8810 women who got their first marriage were included in this study from nine regional states and two administrative cities. Among the total women, 6652 (75.5%) of them gave birth while 2158 (24.5%) of them did not give birth until the end of the interview. Most of the women 6733 (76.4%) lived in a rural, while 2077 (23.6%) lived in urban. The wealth index of the family was categorized as poor, middle, and rich. 4059 (46.1%), 1249 (14.2%), and 3502 (39.7%) women were reported to be from poor, middle, and rich households, respectively. More than half of the women (68%) have not had current work. 61.5% of the total women were uneducated while 38.5% of them were attaining primary and above education level. Furthermore, 4459 (50.6%) of the women had the experience using contraceptive methods while 4351 (49.4%) of them had no experience of using a contraceptive. Regarding exposure to the media, 6280 (71.3%) of the women had no access to mass media and 2530 (28.7%) of them had access to mass media.

### 3.2. Survival Analysis Using Nonparametric Parameters

#### 3.2.1. The Kaplan-Meier Estimate of Time to First Birth of Married Women

To depict the survival of Ethiopian women's time to first birth at varying degrees of the covariate, a nonparametric survival analysis is necessary. It also explains the structure of the survival and hazard functions in the first birth interval dataset. A visualization of the KM curves for survival and hazard experience from time to first birth is shown in Figure 3. At first, the survival plot drops at a rising rate and then decreases at a decreasing rate. This indicates that the majority of women gave birth to their first child soon after marriage. Ethiopian women have a median survival period of 24 years after marriage for their first child (95% CI; 23.4, 25.3).

### 3.3. Comparison of the Different Covariates in terms of Survival Time

To compare the differences between each categorical variable, a formal test was performed using the log-rank test. According to the results of the log-rank test (Table 3), there is a statistically significant difference in the survival experience between the levels of each covariate.

### 3.4. Parametric Shared Frailty Model Results

As a baseline distribution, we used several parametric models with and without gamma shared frailty distributions to fit the data. The model with the lowest AIC and BIC is the best. The results showed that the Weibull-gamma shared frailty model was the best fit for the data (Table 4).

### 3.5. Bayesian Weibull-Gamma Shared Frailty Model Results

The Gibbs sampler algorithm was used to construct parameter inferences, and it was implemented using 20,000 iterations in two separate chains; then, 1,000 terms were removed due to the burn-in state to avoid autocorrelation, and 42,000 samples were collected for the whole posterior distribution. We used a baseline distribution of the Weibull parametric model with and without gamma shared frailty distribution to fit the data. The model with the lowest DIC value is the most suitable. The results revealed that the best model to represent the data was Weibull-gamma shared frailty (Table 5). In this model, frailty is assumed to follow a gamma distribution with a mean of one and a variance of *σ*^2^. Table 5 shows the results of the Weibull-gamma shared frailty model, which reveals that *σ*^2^ = 0.95 suggests regional heterogeneity.

Table 6 shows that all parameter estimates have a Monte Carlo error (MC error) value of less than 5% of the standard deviation, indicating that the parameters are converging. The researcher uses this posterior summary as the final results because of this rationale and convergence graphs. The hazard ratio and 95 percent credible interval of Bayesian technique calculated values were used to analyze the final model findings. At the 5% level of significance, the confidence intervals of the mean for covariates that do not include 0 are significant.

Women who have never used contraceptives have *e*^0.1134^ = 1.12 times increased hazard of first birth (95% CI: 0.06222, 0.1643) than women who have ever used any contraceptive method. Similarly, a researcher can say that the credible interval for the Bayesian hazard ratio did not include the one by exponentiation of the Bayesian credible interval (HR = *e*^0.1134^ = 1.12, 95% CI: *e*^0.06222^, *e*^0.1643^). The risk of first birth among rural residents was increased by 23.5% (HR = *e*^0.2112^ = 1.235) with 95% CI (1.15, 1.33) compared to urban residents keeping other variables constant.

Women who have married 18-34 years have *e*^−1.385^ = 0.25 times decreased hazard of first birth (95% CI: 0.24, 0.26). And those who have married greater than 34 years have *e*^−2.864^ = 0.0561 times decreased hazard of first birth at an earlier age than individuals who married at age less than18 years keeping other variables constant. The husband's education level also affects the timing of the first birth. The hazard of the first birth at an earlier age among married women whose husbands have a primary level of education was increased by 11% (HR = *e*^0.09979^ = 1.11, 95% CI: 1.047, 1.17), and that among married women whose husbands have secondary or above education level was increased by 73% (HR = *e*^0.1148^ = 1.123, 95% CI: 1.04, 1.21) when compared to uneducated husbands keeping other covariates constant. The hazard of the first birth among educated married women was increased by 20% (HR = *e*^0.1826^ = 1.20, 95% CI: 1.15, 1.27) when compared to uneducated women keeping other variables constant.

The estimated coefficient of the parameter for married women who get access to the media was -0.1168. The sign of the coefficient was negative, implying a decreased hazard rate for time to the first birth than those who did not (reference group). The other important variable in this study is the sex of the head of the household. That is, the risk of the first birth among married women whose household head is female was decreased by 16% (HR = *e*^−0.1682^ = 0.845, 95% CI: 0.798, 0.894) when compared to male household heads keeping other variables constant.

### 3.6. Assessment of Convergence

#### 3.6.1. History Plot

The posterior history plots (Figure 4) showed that for 20,000 iterations for each covariate, the model is converging, because the history plot seems tight and able to respond to all parameters.

#### 3.6.2. Density Plot

Figure 5 shows the density plots associated with the coefficient of some selected covariates. Estimates for all parameters revealed good results because the density plot tends to smooth shape.

#### 3.6.3. The Brooks-Gelman-Rubin (BGR) Statistics

The BGR convergence diagnostic graphs in Figure 6 show the line converted into one for stability indicating the convergence of the algorithm.

## 4. Discussion

The major objective of this study was to use Bayesian parametric shared frailty models to find determinant factors for married women's time to first birth in Ethiopia. Ethiopian women had a median survival time of 24 years after marriage for their first child (95 percent CI; 23.4, 25.3). The AIC and BIC criteria were used to compare the model distributions, with the model with the lowest AIC and BIC being accepted [37]. MCMC iteration is used to start the Bayesian approach parametric survival analysis until all parameters have converged. Because there is no known way for choosing an acceptable number of iterations and burn-in size, the MCMC iterations were generated by setting the initial values and burn-in state with no criterion. Rather, the researcher uses a trial-and-error method with the ultimate goal of obtaining stable parameter estimates with the lowest possible simulation error [38]. MCMC simulation improved the accuracy of the results by reducing the credibility interval and lowering the standard error but had no effect on the direction of the results [39, 40]. The Gibbs sampler algorithm of the MCMC iteration method was used to create 42,000 samples in this investigation. 1,000 samples were utilized for the burn-in state, and 20,000 samples with two chains were used for posterior inference utilizing the WinBUGS program for iteration and parameter convergence checks. Weibull distributions with and without the frailty term were compared using the DIC value after the parameters had converged, and the distribution with the smaller DIC value was preferred, as stated by Spiegelhalter [34].

In this study, the Bayesian Weibull-gamma shared frailty model revealed that residence, media exposure, women's education level, husband's education level, contraceptive use, and sex of the household head are statistically significant for married women's survival time to first birth in Ethiopia. This is in line with the findings of a study published in [41, 42].

One of the factors of time to first birth, according to our findings, was one's place of residency. Married women in rural areas have a worse chance of surviving than married women in cities. This is in line with studies [1, 20]. One explanation could be that metropolitan women are more likely to be educated and well informed about contraception use and the consequences of early childbearing [43, 44]. Women who used the contraceptive had a long time to first birth than the nonusers [42, 45, 46]. This is due to the contraceptive service, which helped them in preventing early and unplanned pregnancy throughout their marriage. Age at the first childbirth was also linked to age at marriage. Females who married young had their first child sooner than women who married later. This conclusion is supported by research conducted both domestically and internationally [41, 47, 48]. The reason for this could be that older women need to have a baby shortly after marriage to have the necessary number of children before their reproductive lives come to an end. A woman who marries young can use a contraceptive to delay her first child until she is physically and psychologically mature.

A higher level of education shortens the timing of the first birth after marriage, which is consistent with the findings of [20, 49–51]. Women with a greater level of education had a shorter first birth interval. The link between schooling and the length of the first hiatus from childbearing appears to be indirect. In Ethiopia, increasing women's educational levels is linked to increased labor force participation, media access, and social standing [52]. High levels of education limit parents' traditional roles in deciding on their daughters' marriage partners and encourage self-selection of spouses, which sometimes takes longer. Highly empowered women are, indeed, more likely to have control over not only who and when they marry but also when they have children. This social empowerment of women and the lengthy process of spousal selection are believed to strengthen the intimacy of marriage partners and thus allow them to build strong confidence in each other, which, in turn, increases their desire to have a child to maximize marital satisfaction, resulting in shorter first birth intervals [53]. Furthermore, education improves marital stability by providing stable financial resources. This is also thought to minimize the first birth interval, as they are emotionally ready, biologically mature, and financially comfortable to have a child when they enter married life. In this study, media exposure was found to be inversely related. This is in line with previous research [16, 54, 55]. That is, women who have access to the media had a longer survival period for their first child after marriage. Different advertisements and education about the dangers of early marriage and early childbirth can reduce early marriage and sexual experience and improve understanding of reproductive health issues, which could explain the inverse relationship between media exposure and motherhood at a young age [56]. Women who do not have access to the media, on the other hand, lack adequate awareness of the high-risk period of becoming pregnant and are unaware of family planning options and the costs of early childbearing on the health of mothers and children [57].

### 4.1. Strengths and Limitations of This Study

Although the EDHS is a sizable, nationally representative dataset, this research may have some drawbacks. First, recall bias might be present since survey participants were asked to recall things that happened five years ago, and they might have forgotten some specifics. A second drawback of the data is its cross-sectional design, which makes it challenging to establish causal links between exposure and outcome variables. Third, this study relies on self-reported data from life histories obtained from a nationally representative survey, which is prone to a number of sources of error. As a result, estimates for particular countries may be impacted by these limitations over time, and these should be treated with caution.

While acknowledging these limitations, the EDHS is a nationally representative dataset and has been rigorously designed and deployed by the Centers for Disease Control and Prevention using a global framework, and therefore, the findings can easily be generalized throughout the country. International comparisons of the findings will also be possible because DHSs adopt similar instruments across countries. We anticipate that the findings of this study will have strong policy implications for Ethiopia at the national level, as this is a study that has identified determinant factors of time from birth to first birth.

## 5. Conclusion

The Bayesian method parametric survival model was used to show the determinants of time to first birth among married women in Ethiopia. Based on the DIC value, the Weibull baseline distribution with the gamma shared frailty model was chosen as the best model and the Weibull gamma shared frailty distribution was chosen as the final model to suit the time to first birth dataset. As a result, the results of the Bayesian approach and Weibull AFT model analysis revealed that residence, media exposure, women's education level, husband's education level, contraceptive use, and household head's sex are statistically significant for married women's survival time to first birth in Ethiopia. To curb Ethiopia's rapid population growth, it is necessary to teach families how to use contraception and to raise awareness among rural populations about the importance of increasing the length of the first birth gap and not encouraging early marriage. In general, attempts to reduce fertility by extending the age at first marriage must take into account the socioeconomic and cultural contexts in which marriage takes place. On the other hand, the fight against early marriage should not just focus on reducing reproduction but also on the sociocultural, physiological, and psychological consequences. The impacts of early marriage on the contribution of late marriage to completed family size, on the other hand, need to be investigated further.

## Figures and Tables

**Figure 1:** Sample selection scheme.

**Figure 2:** A graphical illustration of the Bayesian frailty model. Note: *∧*_0_ is the baseline distribution parameter, *β* is the regression parameter of each covariate, *Z* is the frailty distribution, and *θ* is the hyperparameter which follows a gamma distribution.

**Figure 3:** Survival and hazard functions of time to first birth after marriage are plotted using the K-M method.

**Figure 4:** Convergence checking for different covariates.

**Figure 5:** Posterior density for different parameters.

**Figure 6:** Estimated predictive BGR diagnostic graph associated with the coefficient of the covariate.

**Table 1:** List of covariates included in the study.

Variables	Descriptions
Current working of respondents	Yes, no
Age at the first marriage	Women's age when she married (in years)
Region	Tigray, Afar, Amhara, Oromia, Somali, Southern Nations Nationalities and People (SNNP), Benishangul-Gumuz, Gambela, Harari, Addis Ababa, and Dire Dawa are categories of the region
Contraceptive use	Use of contraceptive categorized as yes and no
Media exposure	No, yes
Head of the household	Male, female
Mother's education level	No education, primary, secondary or higher
The highest education level of the husband	No education, primary, secondary or higher
Residence	Urban or rural
Wealth index	Poor, middle, and rich

**Table 2:** Sociodemographic characteristics by time to first birth of married women in Ethiopia (EDHS 2016).

Variables	Categories	Ever given birth by married women	
		Censored no. (%)	Event no. (%)
Region	Tigray	184 (8.5%)	668 (10.0%)
	Afar	136 (6.3%)	617 (9.3%)
	Amhara	290 (13.4%)	711 (10.7%)
	Oromia	261 (12.1%)	962 (14.5%)
	Somali	150 (7.0%)	752 (11.3%)
	Benishangul	183 (8.5%)	550 (8.3%)
	SNNPR	267 (12.4%)	867 (13.0%)
	Gambela	159 (7.4%)	480 (7.2%)
	Harari	128 (5.9%)	382 (5.7%)
	Addis Ababa	231 (10.7%)	323 (4.9%)
	Dire Dawa	169 (7.8%)	340 (5.1%)

Place of residence	Urban	746 (34.6%)	1331 (20.0%)
	Rural	1412 (65.4%)	5321 (80.0%)

Respondent's educational level	No education	1338 (62.0%)	4079 (61.3%)
	Primary	524 (24.3%)	1767 (26.6%)
	Secondary or above	296 (13.7%)	806 (12.1%)

Wealth index	Poor	700 (32.4%)	3359 (50.5%)
	Middle	287 (13.3%)	962 (14.5%)
	Rich	1171 (54.3%)	2331 (35.0%)

Husband/partner's education level	No education	1020 (47.3%)	3130 (47.1%)
	Primary	603 (27.9%)	2158 (32.4%)
	Secondary or above	535 (24.8%)	1364 (20.5%)

Respondent currently working	No	1233 (57.1%)	4770 (71.7%)
	Yes	925 (42.9%)	1882 (28.3%)

Contraceptive use	No	997 (46.2%)	3354 (50.4%)
	Yes	1161 (53.8%)	3298 (49.6%)

Age at the first marriage	Less than 18	1443 (66.9%)	4070 (61.2%)
	18-34	707 (32.8%)	2575 (38.7%)
	Greater than 34	8 (0.4%)	7 (0.1%)

Household head	Male	1716 (79.5%)	5444 (81.8%)
	Female	442 (20.5%)	1208 (18.2%)

Media access	No	1349 (62.5%)	4931 (74.1%)
	Yes	809 (37.5%)	1721 (25.9%)

**Table 3:** Comparison of survival time for time to first birth among married women in Ethiopia (EDHS 2016).

Variables	Categories	Ever given birth by married women			
		Censored no. (%)	Event no. (%)	Log-rank test	*P* value
	Amhara	290 (13.4%)	711 (10.7%)	508.74	≤0.001
	Oromia	261 (12.1%)	962 (14.5%)		
	Somali	150 (7.0%)	752 (11.3%)		
	Benishangul	183 (8.5%)	550 (8.3%)		
	SNNPR	267 (12.4%)	867 (13.0%)		
	Gambela	159 (7.4%)	480 (7.2%)		
	Harari	128 (5.9%)	382 (5.7%)		
	Addis Ababa	231 (10.7%)	323 (4.9%)		
	Dire Dawa	169 (7.8%)	340 (5.1%)		

Place of residence	Urban	746 (34.6%)	1331 (20.0%)	549.66	≤0.001
	Rural	1412 (65.4%)	5321 (80.0%)		

Respondent's educational level	No education	1338 (62.0%)	4079 (61.3%)	335.38	≤0.001
	Primary	524 (24.3%)	1767 (26.6%)		
	Secondary or above	296 (13.7%)	806 (12.1%)		

Wealth index	Poor	700 (32.4%)	3359 (50.5%)	396.71	≤0.001
	Middle	287 (13.3%)	962 (14.5%)		
	Rich	1171 (54.3%)	2331 (35.0%)		

Husband/partner's education level	No education	1020 (47.3%)	3130 (47.1%)	242.1	≤0.001
	Primary	603 (27.9%)	2158 (32.4%)		
	Secondary or above	535 (24.8%)	1364 (20.5%)		

Respondent currently working	No	1233 (57.1%)	4770 (71.7%)	107.66	≤0.001
	Yes	925 (42.9%)	1882 (28.3%)		

Contraceptive use	No	997 (46.2%)	3354 (50.4%)	16.78	≤0.001
	Yes	1161 (53.8%)	3298 (49.6%)		

Age at the first marriage	Less than 18	1443 (66.9%)	4070 (61.2%)	2695.2	≤0.001
	18-34	707 (32.8%)	2575 (38.7%)		
	Greater than 34	8 (0.4%)	7 (0.1%)		

Household head	Male	1716 (79.5%)	5444 (81.8%)	39.6	≤0.001
	Female	442 (20.5%)	1208 (18.2%)		


Media access	No	1349 (62.5%)	4931 (74.1%)	296.7	≤0.001
	Yes	809 (37.5%)	1721 (25.9%)		

**Table 4:** Comparison of different models for time to first birth of women in Ethiopia (EDHS 2016).

Information criteria	Models	No frailty	Gamma shared frailty
	Exponential	55011.326	54923.872
	Gompertz	54838.547	54215.673
	Weibull	54239.872	54121.709
AIC	Log-normal	54329.472	54166.986
	Log-logistic	54891.365	54734.601
	Weibull	54341.031	54235.047

BIC	Log-normal	54413.045	54280.324
	Log-logistic	54981.105	54789.231
	Exponential	55145.892	55003.671
	Gompertz	54976.845	54989.673

**Table 5:** Comparison of models using Bayesian approach for time to first birth of women in Ethiopia, EDHS 2016.

Models	*D*_*bar*_	*D*_*hat*_	PD	DIC
Standard Weibull	45151.000	45127.700	23.300	45174.300
Weibull with gamma frailty	45050.000	45027.800	22.138	45072.100

**Table 6:** Posterior summary for Bayesian Weibull-gamma shared frailty model parameter estimates.

Node	Level of covariates	Mean	MC error	Median	95% CI	Start	Sample
Contraceptive use	Yes	Ref					
beta.co	No	0.1134	6.12*E* − 4	0.1133	(0.06222, 0.1643)^∗^	1001	42000
Residence	Urban	Ref					
beta.rs	Rural	0.2112	0.001564	0.2107	(0.1392, 0.2837)^∗^	1001	42000
Age at the first marriage	Less than 18	Ref					
beta.aam [2]	18-34	-1.385	4.416*E* − 4	-1.386	(-1.434, -1.336)^∗^	1001	42000
beta.aam [3]	Greater than 34	-2.864	0.001607	-2.853	(-3.415, -2.372)^∗^	1001	42000
Current working	No	Ref					
beta.cw	Yes	0.005898	4.918*E* − 4	0.00596	(-0.04255, 0.05403)	1001	42000
Husband education level	No education	Ref					
beta.he [2]	Primary	0.09979	2.699*E* − 4	0.09976	(0.04606,0.1549)^∗^	1001	42000
beta.he [3]	Secondary or above	0.1148	4.314*E* − 4	0.1147	(0.03888, 0.1893)^∗^	1001	42000
Mother education level	No education	Ref					
beta.me [2]	Primary	0.1826	2.77*E* − 4	0.1826	(0.1272,0.2382)^∗^	1001	42000
beta.me [3]	Secondary or above	-0.05222	5.384*E* − 4	-0.0524	(-0.1443, 0.03961)	1001	42000
Media exposure	No	Ref					
beta.mx	Yes	-0.1168	6.564*E* − 4	-0.1168	(-0.174,-0.0585)^∗^	1001	42000
Sex of household head	Male	Ref					
beta.shh	Female	-0.1682	6.217*E* − 4	-0.1681	(-0.2243, -0.1124)∗	1001	42000
Wealth index	Poor	Ref					
beta.wi [2]	Middle	-0.05626	2.698*E* − 4	-0.0563	(-0.1243, 0.01043)	1001	42000
beta.wi [3]	Rich	-0.00962	5.832*E* − 4	-0.0094	(-0.07248, 0.05302)	1001	42000
beta0	Constant	-17.75	0.06547	-17.99	(-18.56, -14.32)^∗^	1001	42000
*R*	Shape parameter	6.097	0.001939	6.097	(6.02, 6.175)^∗^	1001	42000
Sigma	Frailty	0.95	0.001035	0.9988	(0.9483, 1.044)^∗^	1001	42000

Sd = standard deviation; MC error = Monte Carlo error; Ref = reference; 95% CI =95% confidence interval. ^∗^Significant.

## Data Availability

The dataset and supporting materials will be obtained from the corresponding author on a reasonable request.

## Abbreviations

DIC: Deviance information criterion
AIC: Akaike information criterion
BIC: Bayesian information criterion
CSA: Central Statistical Agency
EDHS: Ethiopia Demographic and Health Survey
HR: Hazard ratio
WHO: World Health Organization.
